# Life-History Consequences of Chronic Nutritional Stress in an Outbreaking Insect Defoliator

**DOI:** 10.1371/journal.pone.0088039

**Published:** 2014-02-05

**Authors:** Enric Frago, Éric Bauce

**Affiliations:** Université Laval, Faculté de foresterie et de géomatique, Québec, Canada; CNRS, Université de Bourgogne, France

## Abstract

Food shortage is a common situation in nature but little is known about the strategies animals use to overcome it. This lack of knowledge is especially true for outbreaking insects, which commonly experience nutritional stress for several successive generations when they reach high population densities. The aim of this study is to evaluate the life history consequences of chronic nutritional stress in the outbreaking moth *Choristoneura fumiferana.* Larvae were reared on two different artificial diets that emulate nutritional conditions larvae face during their natural population density cycle (low and medium quality artificial diets). After four generations, a subset of larvae was fed on the same diet as their parents, and another on the opposite diet. We explored larval life-history strategies to cope with nutritional stress, its associated costs and the influence of nutritional conditions experienced in the parental generation. We found no evidence of nutritional stress in the parental generation increasing offspring ability to feed on low quality diet, but the contrary: compared to offspring from parents that were fed a medium quality diet, larvae from parents fed a low quality diet had increased mortality, reduced growth rate and reduced female reproductive output. Our results support a simple stress hypothesis because the negative effects of malnutrition accumulated over successive generations. Density-dependent deterioration in plant quality is thought to be an important factor governing the population dynamics of outbreaking insects and we hypothesize that chronic nutritional stress can be a driver of outbreak declines of *C. fumiferana,* and of forest insects in general.

## Introduction

Resources are frequently limited in natural ecosystems and animals usually face periods of food shortage or are forced to feed on food of suboptimal quality. Many insect species commonly experience chronic nutritional stress and we are now starting to understand the possible strategies used to overcome this situation [1]–[4]. Knowledge on these strategies, however, is still limited for outbreaking insects which commonly experience nutritional stress during several successive generations when they reach high population densities. During outbreaks, massive herbivory leads to food limitation as good quality foliage is depleted and host plant productivity is reduced. Even with abundant foliage, herbivory can lead to reduced plant nutritional quality [5] because insect feeding commonly elicits a wide variety of induced plant defences aimed at deterring or reducing it (reviewed in [6], [7]). Understanding insect outbreaks is an area of intense debate in insect-plant interactions. Based on empirical and theoretical work it has been hypothesised that population cycles are strongly governed by herbivore-induced density-dependent deterioration in plant quality [8]–[13]. Using small-scale laboratory experiments, the life history strategies employed by insects to cope with nutritional stress can be assessed (e.g. [1]), and this information can be valuable to understand long-term population dynamics, for example by improving parameterisation of theoretical models [12].

By experimentally manipulating food quality for several consecutive generations, the potential for a species to develop plastically as a response to chronic nutritional stress can be tested in the laboratory (e.g. [1]). Plastic responses are expected to be favoured over specialisation in heterogeneous environments (e.g. [14], [15]), and this is likely to be a common strategy for outbreaking species in response to variation in food quality or availability. In insect species with non-feeding adults, or whose adults feed very little, plastic responses occur at the larval stage through physiological changes [16] and plasticity in life-history traits [17], [18]. Larval plastic responses, however, are usually traded-off against adult traits and adults can exhibit reduced survival, reproduction or dispersal; costs can even carry over the next generation through maternal effects [19]. Despite much attention having been paid to insect life histories and insect responses to nutritional stress in model species, responses to chronic nutritional stress in outbreaking insects remains relatively unexplored.

We used as a model system the spruce budworm, *Choristoneura fumiferana* Clemens (Lepidoptera: Tortricidae). This boreal moth commonly outbreaks and is the most economically important forest insect pest in north-eastern North America [20], [21]. *C. fumiferana* larvae feed on foliage of balsam fir, *Abies balsamea,* of varying nutritional quality. During outbreaks, high quality current-year foliage of the upper crown may become depleted and larvae must feed on either one-year-old foliage or lower crown foliage which are of suboptimal quality [22], [23]. *C. fumiferana* outbreaks usually last between five to eight years [24], as a result outbreaking populations need to develop and successfully reproduce under nutritional stress for several successive generations. The causes of outbreak declines in this species, and in forest pests in general, are poorly understood with some evidence suggesting that nutritional quality might be a contributing factor. After several consecutive years of *C. fumiferana* defoliation, balsam fir foliage has increased amounts of raw fibre which negatively affects *C. fumiferana* development and survival [25]. Trans-generational effects are also likely to magnify chronic nutritional stress as parental nutritional stress carries over to the next generation: in the laboratory *C. fumiferana* parents that were fed low quality food laid few viable eggs and their offspring had increased mortality [26], [27]. Similarly, females mated with males that fed on a low quality diet had reduced fecundity [28].

Here, we used artificial diets to emulate the nutritional conditions *C. fumiferana* larvae experience during the natural population density cycle. We tested the hypothesis that larval populations will show increased ability to feed on low quality diet within four generations. We also tested whether this was traded-off against feeding on medium quality diet. Under the adaptation maternal hypothesis [29]–[31] the nutritional conditions experienced by parents will induce changes in the offspring that will increase their fitness under the same conditions. A simple stress hypothesis would otherwise predict that offspring whose parents were fed a low quality diet will have reduced fitness on both diets as compared to offspring from parents that were fed a medium quality diet. To gain a deeper understanding of the traits involved in these responses, several life history parameters were measured including mortality, several larval development traits and female reproductive output.

## Materials and Methods

### Artificial Diets

During the first generation of the study, larvae were reared on three diet types: low, medium and high quality diets. The high quality diet was the standard McMorran’s diet [32] which provides optimal growth and development of *C. fumiferana* larvae in the laboratory and contains 5.6% nitrogen and 23% soluble sugar. The other two were created following Bidon’s method [33]: the medium quality diet contained 5% nitrogen and 12% soluble sugar, and the low quality diet contained 7% nitrogen and 1.5% soluble sugar. For the following generations, we limited the number of diets tested to those two that best emulated the nutritional conditions that larvae experience in nature during the dynamic population density cycle. We chose the medium and low quality diets over the standard McMorran’s diet because the nutritional conditions they provide lead to insect performances similar to what is found in natural populations, or when larvae feed natural foliage. When feeding on McMorran’s diet, for example, larval mortality is commonly lower than 30% whereas on natural foliage average mortality is 50% [34]–[36].

### Insect Rearing

Larvae were supplied by the Forest Pest Management Institute, Forestry Canada (Sault Sainte-Marie, Ontario) and were reared on standard McMorran’s diet [32] for four successive generations before the start of the experiment. Larvae were reared at 23°C, 65% r.h. and L16:D8 photoregime in 30 ml clear plastic containers filled with a thin layer of artificial diet (two larvae per container). Once larvae pupated, and the adults emerged one male and one female belonging to the same treatment but from different maternal lines were placed in a clear plastic vial (9.5 cm high x 4.5 cm in diameter) with the top covered by a piece of cheesecloth. Moths were fed daily with sugar solution. Throughout the oviposition period the eggs laid by each female were collected every other day. Eggs were placed in clear plastic boxes (4×2.5×1.5 cm) whose lids were lined with cheesecloth in order to provide a place for the first instar larvae to build hibernacula. Eggs were incubated in the same conditions as larvae. Once larvae built hibernacula, winter conditions for diapause were emulated following [37].

### Experimental Design

Larvae were fed on low and medium quality diet for four generations starting from a total of 800 post-diapausing larvae representing the offspring of 65 different females. Each generation took one year so that the whole experiment lasted for four years. This type of experiments usually include contemporary replicated lines within each treatment [38], but due to technical constraints, a single line per diet type was maintained. To correct for this, analyses were conducted by fitting generalized animal models (see statistical analyses for further details). Also due to the large amount of time required to rear the insects, only 400 randomly selected post-diapausing larvae per generation and treatment were maintained. In the fourth generation, larvae from both diet types (hereafter referred to as parental diet) were randomly split into two groups and reared on the original as well as the opposite diet (hereafter referred to as offspring diet). Insect development in the fourth generation was monitored daily by recording larval mortality, the date of pupation and of adult emergence. Pupae were weighted to the nearest 0.1 mg and sexed within 24 h of pupation. Four weeks after oviposition, eggs as well as live offspring were counted.

### Variables Measured

For each individual the following variables related to larval development were measured. (i) survival from second instar to adulthood. (ii) Pupal weight. (iii) Development time from second instar larvae to imago emergence. (iv) The exponential growth rate over the post-diapausing larval period was calculated in order to express how efficiently the time available was used to gain adult mass [1]. Growth rate was estimated by calculating the logarithm of pupal weight divided by egg weight and this was then divided by development time from post-diapausing second instar larvae to imago emergence. Egg weight was obtained from [26] and was fixed at 0.21 mg, and was used as a proxy for post-diapausing second instar larval weight as pre-diapausing *C. fumiferana* larvae do not feed [21]. The following variables related to female reproductive output were also measured. (i) Female fertility was estimated by considering each coupled female as fertile when she laid at least one viable egg. For each fertile female (ii) realized fecundity, as the number of eggs laid, and (iii) fecundity, as the number of viable eggs, were also estimated.

### Statistical Analyses

All analyses were performed in R 3.0.1 (http://www.r-project.org/). In the first generation, the effect of low, medium and high quality diet on larval development traits and also on female realized fecundity and fecundity were tested with ANOVA followed by a post-hoc test performed with the *testFactors* command in the *Phya* package. For larval development traits males and females were analysed independently. Differences in mortality and in the proportion of fertile females were evaluated with a generalized linear model assuming a quasibinomial error distribution.

Analyses in the fourth generation were conducted by fitting generalized animal models for each life history trait studied. An animal model is a type of mixed effects model where, in addition to any other fixed or random effect, an individual’s phenotype is a function of the resemblance among individuals. Such resemblance is included in the model in the form of a pedigree, or a random additive genetic “animal” effect [39], [40]. The reason for using this approach is that, due to technical constraints, a single line of insects was studied on each diet type so that any differences among individuals in the two different parental diets could exclusively be due to genetic drift. By adding an “animal” random effect in the models this can be accounted for [39], [40]. Animal models were fitted with Bayesian Markov chain Monte Carlo (MCMC) techniques implemented in the MCMCglmm package [41]. A crucial step when using Markov chain Montecarlo techniques is the choice of appropriate priors. We ran the MCMCglmm for 1×10^7^ iterations modifying the default priors to allow optimal mixing of the chains and weak autocorrelations among subsequent iterations. Fixed effect priors were drawn from the normal distribution with mean = 0.002 (gaussian models) or mean = 0.99 (bivariate models) and variance = 1000. Random effects priors were set at variance = 1 and degree of belief = 1. For the fixed effect priors other values were also tested and lead to similar results. To prevent autocorrelation among subsequent iterations the chain was sampled every 4500 iterations and the first 1×10^6^ iterations were removed as burn-in. Autocorrelation between consecutive values was low (<0.1), there were no trends in the chain and posterior distributions were not skewed.

All models were built with a gaussian response, except mortality and female fertility which were built with a bivariate response (i.e. dead vs. alive or fertile vs. non fertile female). For each trait studied a set of models was built including the null model, parental and offspring diet as fixed factors, sex (only in the models for larval development traits) and their pairwise interactions. To evaluate the importance of each term we used an information theoretic approach [42] using the deviance information criterion (DIC) in the MCMCglmm package [41], [43]. DIC has a similar behaviour than the Akaike Information criterion [44] so that the model with the smaller value can be considered as the best model DIC_min_ [42]. Each model in the set can then be ranked according to its difference in the DIC score in comparison to DIC_min_. Model weight (w) was also calculated for each model as a measure of evidence in favour of each model being the best within the set. Model selection was achieved by selecting a 95% confidence set of models with a cumulative DIC weight of 0.95 (i.e. a 95% confidence that the best model was selected, [42], [45]). As a conservative measure, when for a specific trait the 95% confidence set of models included the null model, all fixed terms or interactions were considered to have a negligible effect on the response.

## Results

### Direct Effects of Diet Quality

In the first generation larvae reared on high quality diet suffered less mortality than those reared on low quality diet (Logistic regression; χ^2^_2df = _2.72; *P* = 0.0066), but mortality was not significantly different from those reared on the medium quality diet (Logistic regression; χ^2^_2df = _1.12; *P* = 0.2639; Fig. 2). All measured larval development traits were affected by diet type in both sexes (Fig. 1): female pupal weight: *F*_2,43_ = 13.53, *P*<0.0001; male pupal weight: *F*_2,59_ = 14.79, *P*<0.0001; female development time: *F*_2,43_ = 11.00, *P*<0.0001; male development time: *F*_2,59_ = 5.85, *P* = 0.0048; female growth rate: *F*_2,43_ = 13.90, *P*<0.0001; male growth rate: *F*_2,59_ = 10.52, *P* = 0.0001. The post-hoc test (Fig. 1) revealed that larvae reared on medium or high quality diets showed no differences in the larval developmental traits measured, but larvae reared on low quality diet developed into smaller pupae, spent more time from second instar to adulthood and had a lower growth rate. In mated females, the probability of laying at least one fertile egg was not significantly different among females reared on the different diets (Logistic regression; *F*_2,31_ = 0.23 *P* = 0.7961). Among fertile females, diet type did not affect female realized fecundity (*F*_2,19_ = 1.60; *P* = 0.2279) or fecundity (*F*_2,19_ = 1.69; *P* = 0.2110) (Fig. 2).

**Figure 1:** *Choristoneura fumiferana* larval development traits in the first generation. Mean pupal weight, development time and growth rate (±SE) of larvae feeding on high (grey), medium (white) and low (black) quality diet. The first three bars in each graph represent larval development traits for females and the other three represent males’ traits. Also shown is the number of larvae per treatment or sex. Bars belonging to the same sex with the same letter on the top do not differ significantly (p<0.05).

**Figure 2:** *Choristoneura fumiferana* female reproductive output and mortality in the first generation. Mean realized fecundity and fertility (±SE), proportion of fertile females and proportion of dead larvae on high (grey), medium (white) and low (black) quality diet. Also shown is the number of larvae used to estimate realized fecundity and fertility in each treatment.

### Effect of Parental and Offspring Diet

Most of the traits studied were influenced by the explanatory variables included in the models (Fig. 3, 4 and Table 1). In the models for mortality, the interaction between parental and offspring diet was the only term included (Table 1). Mortality was lower on a medium quality diet with no differences associated to parental diet, but on a low quality diet nutritional stress in the parental generation lead to increased levels of mortality (Fig. 4). In the models for pupal weight only the interaction term between offspring diet and sex was included in the confidence set (Fig. 3 and Table 1). Larvae reared on low quality diet developed into lighter pupae, but the effect was stronger in males (weight loss was 33.9% for males and 24.7% for females). Two models were included in the 95% confidence set of models for development time. The interaction term between parental and offspring diet had the higher model weight (0.65) followed by the interaction term between offspring diet and sex (0.31). Larval development took longer in females as well as in larvae whose parents were fed a low quality diet, but these differences were less evident when larvae were fed a low quality diet. For growth rate, offspring diet as fixed term was included in the subset of models as the variable with higher weight (0.78), larvae on low quality diet showed lower growth rate. The models for growth rate also included the interaction term between offspring diet and sex (0.15), and the interaction between offspring and parental diet (0.07). The phenotypic response reveals that although the sex of the individual and the parental diet influenced growth rates, these effects were almost unnoticeable when larvae were fed a low quality diet. In the models for fertility (i.e. probability of a mated female to lay at least one fertile egg) both parental and offspring diet were included in the confidence set with model weights of 0.22 and 0.20, respectively. The interaction term between these two fixed factors had the higher weight (0.53), and the phenotypic response reveals that the lower probability to develop into a fertile female was recorded when larvae whose parents were fed a low quality diet were also fed this same diet. For those females that laid at least one viable egg, the 95% confidence set included the null model in the models with female realized fecundity (number of eggs) and female fecundity (number of viable eggs) as response. This suggests that diet had a negligible effect on these two traits.

**Figure 3:** *Choristoneura fumiferana* larval development traits of lines feeding on medium and low quality diet for four generations and then fed the same and the opposite diet. Mean pupal weight, development time and growth rate (±SE) of females whose parents (i.e. parental diet) fed medium (dark grey) or low (white) quality diet, and males whose parents fed medium (black) or low (light grey) quality diet. The first four bars in each graph represent larval development traits of lines feeding on medium quality diet and the other four represent lines feeding on low quality diet (i.e. offspring diet). Also shown is the number of larvae per treatment and sex.

**Figure 4:** *Choristoneura fumiferana* female reproductive output and mortality of lines feeding on medium and low quality diet for four generations and then fed the same and the opposite diet. Mean realized fecundity and fecundity (±SE), proportion of fertile females and proportion of dead larvae of individuals whose parents (i.e. parental diet) fed medium (grey) or low (white) quality diet. The first two bars in each graph represent traits of lines feeding on medium quality diet and the other two represent lines feeding on low quality diet (i.e. offspring diet). Also shown is the number of larvae used to estimate realized fecundity and fertility in each treatment.

**Table 1:** Effect of offspring and parental diet on *Choristoneura fumiferana* life history traits evaluated with generalized animal models fitted with Bayesian Markov chain Monte Carlo (MCMC) techniques.

wi		Mortality	Pupal weight	Dev. time	Growth rate	Fertility	Relized fecundity	Fecundity
	Parental diet					0.217		
	Offspring diet				0.780	0.196		
	Sex	–				–	–	–
	Par. x Off. diet	0.999		0.646	0.065	0.533		
	Parental diet x Sex	–				–	–	–
	Offspring diet x Sex	–	0.999	0.307	0.154	–	–	–
Σwi		0.999	0.999	0.953	0.999	0.946		
DICi								
	1 st	32.4	2087.4	1546.5	−700.6	2.6	581.0	590.0
	2 nd			1548.0	−697.4	4.4	581.4	593.2
	3 rd				−695.7	4.6	582.3	594.1
	null	65.4	2280.0	1612.7	−684.1	7.2	583.0	594.8

For each trait a set of models was built including the null model, parental and offspring diet as fixed factors, sex (only in the models for larval development traits) and their pairwise interactions. The importance of each term was evaluated using an information theoretic approach with the deviance information criterion (DIC). For each model in the 95% confidence set, weights (w) and the DIC are presented. The DIC for the null model is also presented. Weights for the models for realized fecundity and fecundity are not presented because the 95% confidence set included the null model so that we consider that all fixed terms or interactions had a negligible effect on the response.

## Discussion

The economic importance of outbreaking insects has generated numerous studies addressing how plant nutritional quality affects their fitness [46]. Bioassays commonly focus on a single generation and little is known about the long-term multigenerational effects of diet quality. Our study shows that larvae of the outbreaking moth *C. fumiferana* were affected by diet quality in the first generation, but more importantly, that they are able to survive and successfully reproduce when feeding on low quality food for several successive generations. Chronic nutritional stress affected larval development traits and led to reduced survival and female reproductive output, with no evidence of nutritional stress in the parental generation increasing offspring ability to feed on low quality diet. Our data supports a simple stress hypothesis because relative to offspring of parents that were fed a medium quality diet, larvae whose parents were fed a low quality diet showed increased mortality and reduced female fertility, even when offspring fed on medium quality diet. Nutritional quality in the parental generation also affected larval developmental traits as larvae whose parents were fed a low quality diet had a longer developmental time and a reduced growth rate. Both responses are commonly held as being disadvantageous because a longer development time, or reduced growth rate, might extend the risk of mortality, a phenomenon known as the slow-growth-high-mortality hypothesis [47], [48].

The experiment reported here was designed to produce mild and strong nutritional stress on the larvae. Based on the amount of total nitrogen and soluble sugar, both the medium and low quality diets mimic the nutritional conditions *C. fumiferana* experiences in natural conditions [26]. For example, larvae that were fed a medium quality diet for four generations showed values of mortality, pupal weight, development time and female reproductive output similar to what is found when larvae feed on natural foliage in experimental field stands [34], [35]. Most of our knowledge on the genetic and physiological bases of responses to nutritional stress, and its life history consequences, comes from studies with *Drosophila* [49]. Although *C. fumiferana* life history characteristics posed a limitation to the number of generations and replicated lines used, one of the problems in interpreting results from other model insects is the lack of an appropriate ecological context. Many species, like *Drosophila,* face periods of food shortage but this condition is not commonly extended for several generations. When outbreaking insects reach high densities, however, larvae commonly feed on low quality foliage for several generations. In *C. fumiferana* direct negative effects of defoliation on larval performance [23], [25] as well as on the following generation through maternal effects [26], [27] are well documented. There is increasing recognition from theoretical studies and empirical evidence that density dependent reduction in foliage quality is an important intrinsic cause underlying outbreak declines in insects [8]–[13]. Our results are in agreement with this hypothesis because after four consecutive generations of nutritional stress, survival and female reproductive potential were reduced. Special attention has also been paid on whether density dependent decrease in nutritional quality is mainly dominated by either foliage depletion or by inducible plant defences [12], [13]. However, the limited number of long-term multigenerational studies that have manipulated food quality still hampers our understanding of how plant quality and availability is linked to crashes in insect populations. It would be very exciting to perform long-term experiments manipulating not only nitrogen and sugar content, but also secondary defensive compounds as they are key players in insect-plant interactions.

Not all larval development traits were similarly affected by chronic nutritional stress. Larval developmental time and growth rate were affected but not pupal weight, which suggests that plasticity in larval growth was a plastic response that reduced the impact of parental nutritional stress on pupal size (a trait highly correlated with adult fitness). Since plastic responses are constrained by trade-offs among different growth parameters and fitness components [17], [18], in our study they might be the underlying cause of increased mortality and reduced fertility under chronic malnourishment. The costs of increased larval developmental time in *C. fumiferana* females were also likely to limit plasticity in this trait as nutritional stress usually leads to extended developmental time, but this wasn’t shown by females on low quality diet. An adaptation maternal hypothesis [29]–[31] would predict that the nutritional conditions experienced by parents will induce changes that will benefit the offspring under the same conditions. The increased development time and reduced growth rate in larvae from malnourished parents is in disagreement with this hypothesis and again supports a simple stress hypothesis because extending larval development usually increases mortality risk [47], [48]. Under nutritional stress, reducing the growth rate is also a poor option because low nutritional quality usually signals that conditions will continue to worsen from that moment on. For instance, *Drosophila* lines selected under crowded conditions or under chronic nutritional stress evolved higher feeding rate [49], higher growth rate [1] or a smaller threshold size for pupation [50]. These conditions might signal, for example, an increase in intraspecific competition or reduced suitability of a decomposing fruit. Similar ecological conditions leading to fast nutritional deterioration are also common in outbreaking insects, and increased developmental time or lower growth rate would imply extending malnutrition. Physiological responses to stress in insects are little understood and hormones induced during nutritional stress can affect many different traits (e.g. [51]). Since only few adult life history traits were measured or selected in the present work, it is possible that the reaction norm observed in larval development reflects changes in adult traits not measured here. For instance, allocation decisions can affect flight ability and therefore the females’ ability to choose oviposition sites or for dispersal. In the butterfly *Speyeria mormonia*, nutritional stress altered the allometric relationship between pupal weight and wing span [52] and in *Malacosoma disstria* it shifted allocation in reproduction versus somatic growth [53]. In the butterfly *Bicyclus anynana* malnourished larvae lead to smaller adults but they had increased flight abilities due to body allocation changes [54]. In *Drosophila,* populations selected under nutritional stress evolved behavioural strategies likely to improve foraging efficiency [2], [3]. Several forest pests, and *C. fumiferana* in particular, are known to outbreak in temporal synchrony throughout extensive areas in the landscape, and dispersion is thought to be an important mechanisms behind it (e.g. [55]–[57]). Finding out whether nutritional stress affects allocation decisions that improve the females’ dispersal would help in understanding how outbreaking species exploit their hosts at the landscape level.

In conclusion, our results show that several consecutive generations of nutritional stress have a dramatic effect on performance in the outbreaking moth *C. fumiferana,* especially on survival and the proportion of fertile females. Such a decrease in fitness can be a potential driver of outbreak declines in *C. fumiferana,* but also in other forest insects. Transgenerational effects can also be important in understanding time lags between outbreaking events because even with abundant and good quality foliage, nutritional stress experienced in previous generations can restrict population growth. The life history traits measured here were related to larval development, survival and reproductive output, but nutrition-related transgenerational effects are also likely to affect other important traits. Among them, female dispersal [16], [53], [54] or interactions with higher trophic levels (for example through changes in immune investment, [58]) can be potentially important to understand insect outbreaks at the landscape level, but also from a multitrophic perspective. A substantial amount of theoretical and empirical research has been devoted to understanding how nutritional quality and availability governs the population ecology of outbreaking insects [12], [13] but specific studies to unveil how this is affected by chronic nutritional stress are still lacking.
